This article has been retracted.

# Effect of Bisphenol A-Mediated RBP-4 on Pregnancy Outcomes in Nonobese Pregnant Female with Subclinical Hypothyroidism

**DOI:** 10.1155/2022/9716224

**Published:** 2022-07-20

**Authors:** Danyan Chen, Hongman Wang, Xi Chen, Li Li, Liwei Luo, Rongxi Huang

**Affiliations:** ^1^Departments of Endocrinology, Chongqing General Hospital, Chongqing 401147, China; ^2^Departments of Science & Education, Chongqing General Hospital, Chongqing 401147, China

## Abstract

Hypothyroidism is a systemic hypometabolic syndrome caused by the thyroxine resistance or a reduction in its extent. It is an endocrinopathy secondary to gestational diabetes and occurs usually without significant symptoms. This study explored the effect of bisphenol A (BPA)-mediated retinol-binding protein 4 (RBP-4) on pregnancy outcomes in a nonobese pregnant female with subclinical hypothyroidism. Three hundred nonobese pregnant females who had that established pregnancy files and had regular obstetric examinations from January 2021 to March 2022 were enrolled and classified with 100 cases in each group as early pregnancy (6–12 weeks of gestation), second-trimester (13–24 weeks of gestation), and third-trimester groups (25–36 weeks of gestation). Thirty pregnant women with subclinical hypothyroidism were selected as subjects, and another thirty pregnant women with normal thyroid function were selected as the normal control group. Thyroid function (thyroid-stimulating hormone (TSH), free triiodothyronine (FT_3_), free T_4_ (FT_4_), and thyroid peroxidase antibody (TPO-Ab)) was measured by immunoelectrochemiluminescence. The level of BPA in urine was determined by solid-phase extraction high-performance liquid chromatography-tandem mass spectrometry. Serum RBP4 levels were determined by enzyme-linked immunosorbent assay. The level of TSH in the third-trimester group was higher than that in the first- and second-trimester groups, while the levels of FT_3_, FT_4_, and TPO-Ab were lower than those in the other two groups (*P* *<* *0.05*). TSH in the second-trimester group was higher than that in the first-trimester group, while FT_3_, FT_4_, and TPO-Ab levels were lower than those in the first-trimester group (*P* *<* *0.05*). The levels of BPA and RBP4 in gestational diabetes mellitus and hypertension were higher than those in the nongestational period, and the levels of BPA and RBP4 in gestational intrahepatic cholestasis and anemia were higher than those in the nongestational period, and the levels of BPA and RBP4 in preterm delivery were higher than those in nongestational period (*P* *<* *0.05*). Also, the level of urinary BPA in the hypothyroidism group was higher than that in the normal control group (*P* *<* *0.05*) and the level of serum RBP4 in the hypothyroidism group was higher than that in the normal control group (*P* *<* *0.05*). According to multivariate logistic regression analysis, age ≥30 years and the ascending BPA and RBP4 were risk factors for subclinical hypothyroidism during pregnancy in the nonobese female. BPA and RBP-4 are closely related to the pregnancy outcome of nonobese subclinical hypothyroidism in the pregnant female. The degree of BPA and RBP-4 in adverse pregnancy outcomes is increased, which is the risk factor for nonobese subclinical hypothyroidism.

## 1. Introduction

The thyroid is the largest endocrine gland in the human body, which secretes thyroid hormone to participate in different metabolic activities in human function which can restrict the growth and development of the body. Hypothyroidism is caused by reduced levels of thyroid hormones, which play an important role in the development of bone tissue and in the regulation of energy metabolism in women during pregnancy. However, hypothyroidism during pregnancy can affect the fetus and may cause fetal malformations and mental retardation and, in severe cases, may lead to adverse pregnancy outcomes such as abortion and preterm delivery. Therefore, it is important to screen thyroid function early in pregnancy to diagnose and to provide timely intervention, while at the same time, it is also clear that the influencing factors of hypothyroidism during pregnancy are beneficial to reducing or avoiding adverse pregnancy outcomes and it can also promote fetal development. Thyroid hormone is a growth hormone, which is involved in tissue growth, energy metabolism and protein synthesis. It is more significant in pregnant female and is involved in maternal placenta growth, bone development and fetal nervous system, etc. [1, 2]. The decrease or increase of thyroid hormone level will affect the development of the fetus, resulting in malformation, mental retardation and other adverse pregnancy outcomes such as premature delivery and abortion [3]. Hypothyroidism (hypothyroidism) is a systemic hypometabolic syndrome caused by thyroxine resistance or its reduced degree. It is an endocrine disease secondary to gestational diabetes mellitus and usually has no obvious symptoms [4]. Exposure to Bisphenol A (BPA) during pregnancy not only affects maternal thyroid disease, but also directly causes adverse pregnancy outcomes [5]. Retinol binding protein 4 (RBP-4) is a newly discovered adipocytokine, which is involved in glucose regulation and metabolism and induces insulin resistance [6]. The purpose of this study was to investigate the effect of BPA-mediated RBP-4 on pregnancy outcomes in non-obese pregnant women with subclinical hypothyroidism.

## 2. Data and Methods

### 2.1. General Information

Three hundred nonobese pregnant females who had established pregnancy files and had regular obstetric examinations from January 2021 to March 2022 were enrolled and classified with 100 cases in each group as early pregnancy (6–12 weeks of gestation),second-trimester (13–24 weeks of gestation), and third-trimester groups (25–36 weeks of gestation). Thirty pregnant women with subclinical hypothyroidism were selected as subjects, and another thirty pregnant women with normal thyroid function were selected as the normal control group.

Inclusion criteria: those with complete data of maternal pregnancy examination; aged between 18 and 40; married and naturally conceived with accurate gestational age; no use of antibiotics, immunomodulators, or steroid hormones during pregnancy; and single live fetuses in intrauterine pregnancy.

Exclusion criteria: those with twin or multiple fetuses; ovulation induction or assisted reproductive technology; with thyroid disease, rheumatoid arthritis, systemic lupus erythematosus, and other autoimmune diseases before pregnancy; with hypertension, diabetes, abnormal metabolism of lipoprotein, abnormal parathyroid function, or tumor before pregnancy; with severe organ dysfunction in renal, heart, lung, liver, or systemic diseases; who took medications before or during pregnancy that may affect the thyroid function or have undergone thyroid hormone replacement therapy or thyroid surgery. with adverse pregnancy outcomes of premature pregnancy, abortion, placenta previa, or placental abruption; and cognitive impairment and mental illness before pregnancy, or those who withdrew from the study due to poor compliance.

### 2.2. Criteria for Subclinical Hypothyroidism and Pregnancy Outcomes

Subclinical hypothyroidism: the thyroid-stimulating hormone (TSH) levels in early pregnancy were between 2.5 and 10 mIU/L and the TSH levels in the second and third trimesters was between 2.5 and 10 mIU/L and the level of free T4 (tetraiodothyronine, FT4) was normal. The positive TPO-Ab was excluded to exclude the effect of thyroid peroxidase antibody (TPO-Ab) on pregnancy outcome. The TPO-Ab < 60 U/ml was negative.

Pregnancy outcomes: (1) assess for gestational diabetes: a glucose tolerance test was performed on the subjects at 24–28 weeks of gestation. 75 g of glucose was taken orally. The diagnostic criteria of gestational diabetes are as follows: fasting blood glucose ≥ 5.1mmol/l, blood glucose ≥ 10.0mmol/l 1h after taking sugar, and blood glucose ≥ 8.5mmol/l 2h after taking sugar, one of which can be diagnosed. (2) Assess for hypertensive disorders during pregnancy: if there was no history of hypertension and family history of hypertension before pregnancy, the secondary hypertension was excluded. Those with blood pressure ≥140/90 mmHg and negative urine protein can be diagnosed with gestational hypertension. (3) Assess for intrahepatic cholestasis of pregnancy: if the serum total bilirubin increased and exceeded 68 *μ*mol/L during pregnancy, the elevation of serum bile acid to 10 times normal, alkaline phosphatase activity, and mild to moderate elevation of transaminase can be diagnosed as intrahepatic cholestasis of pregnancy. (4) Assess for anemia in pregnancy: pregnancy anemia can be diagnosed if the peripheral blood hemoglobin level was lower than 110 g/L and the hematocrit was lower than 0.33. (5) Assess for premature birth: preterm birth was diagnosed if the pregnancy reached 28 weeks but delivery was less than 37 weeks.

### 2.3. Determination of Index

#### 2.3.1. Collection of Serum and Urine Samples

5 ml each of maternal urine and fasting venous blood were collected, and the serum was separated by centrifuging venous blood for 10 min at 3000 r/min in a high-speed refrigerated centrifuge (the upper layer is in light yellow or clear color, i.e., serum). The urine and serum samples were immediately stored in a −20°C freezer protected from light and then it was transferred to a−80°C freezer for freezing.

#### 2.3.2. Determination of Thyroid Function Index

The serum samples were collected, and the thyroid function was measured by immunoelectrochemiluminescence with an automatic immune analyzer, including TSH, triiodothyronine (FT3), FT4, and TPO-Ab. Siemens instruments and kits were used.

#### 2.3.3. Determination of Urinary BPA

Urine was measured by solid-phase extraction and high-performance liquid chromatography-tandem mass spectrometry. Add 1 mol/l (pH 6.5) ammonium acetate buffer 500μl , 200 ng/ml mixed bishenol a-d16 (sigma, USA) isotope internal standard working solution 100 μ l, and 200 U/ml β- Glucosidase solution 200 μ l to the centrifuge tube. Enzymolysis at 37 °C for 90min. The urine was cooled to room temperature after enzymolysis. 1 ml of ammonia solution was added to the urine specimen for use. After the max solid-phase extraction column was activated with 3 ml acetonitrile and 3 ml water in turn, the enzymolysis urine sample was loaded through the column at a speed of 1 ml/min, and then the column was washed with 3 ml water and acetonitrile in turn and subsequently dried for 5 min. Finally, 3 ml acetonitrile/ethyl acetate containing 2% formic acid (1 : 1 by volume) was eluted and collected. The eluate was dried under nitrogen at 50°C, reconstituted by adding 200 *μ*l of 20% acetonitrile solution, vortexed for the 30s, and 10 *μ*l of the reconstituted solution was injected for analysis. The internal standard curve method was used for quantitative analysis, and the concentration of the unknown substance was determined by comparing the area ratio of the unknown substance to the internal standard substance and the area ratio of the standard substance to the internal standard substance. The linear correlation coefficient of the standard curve was higher than 0.99, and the limit of detection (LOD) was 0.2 *μ*g/L.

#### 2.3.4. Determination of Serum RBP4

RBP4 expression levels in serum were examined using the ELISA (RayBiotech, Atlanta, USA). Briefly, the standards and the samples to be tested were added to the corresponding wells and then incubated with detection antibodies labeled with horseradish peroxidase. The plate was covered with a sealing film and was incubated in a 37°C water bath for 60 minutes. The reaction solution was discarded, and after washing, the plates were patted dry and then incubated at 37°C with the corresponding substrate for 15 min in the dark. Finally, 50 *μ*L of stop solution was added and within 15 min, the OD value was obtained using a microplate reader (Biorad, Hercules, CA, USA) to a wavelength of 450 nm.

### 2.4. Statistical Treatment

Two people input the data into EpiData 3.0 software, statistical analysis with SPSS 22.0. The measurement data were expressed in ($\bar{x}$ ± *s*) and the *t-*test was adopted; statistical data were expressed as constituent ratios, and the *χ*^2^ test or Fisher test was used for an accurate test. The comparison of three groups or above was by way of ANOVA. The factors of subclinical hypothyroidism during pregnancy in nonobese female were analyzed by logistic regression. The difference was statistically significant (*P* *<* 0.05).

## 3. Results

### 3.1. Comparison of Thyroid Function Levels at Different Stages of Pregnancy

The TSH levels in the third-trimester group were higher than those in the first-trimester and second-trimester groups, while the FT3, FT4, and TPO-Ab levels were lower than those in the first-trimester and second-trimester groups (*P* *<* 0.05); the levels of TSH in the second-trimester group were higher than those in the first-trimester group, while the FT3, FT4, and TPO-Ab levels were lower than those in the first-trimester group (*P* *<* 0.05), as shown in Table 1.

### 3.2. Comparison of Urinary BPA Levels in Different Pregnancy Outcomes

The level of BPA in urine and hypertension of gestational diabetes was higher than that of nongestational diabetes mellitus and hypertension; the urine BPA of intrahepatic cholestasis of pregnancy and anemia was higher than that of nonpregnancy and the level of BPA in preterm urine was higher than that in the nonpreterm labor (*P* *<* 0.05), as shown in Table 2.

### 3.3. Comparison of Serum RBP4 Levels in Different Pregnancy Outcomes

The level of serum RBP4 in gestational diabetes mellitus and hypertension was higher than that in nongestational intrahepatic cholestasis and anemia in pregnancy and premature delivery was higher than that in nongestational anemia (*P* *<* 0.05), as shown in Table 3.

### 3.4. Comparison of Urinary BPA and Serum RBP4 between Hypothyroidism Group and Normal Control Group

The levels of urinary BPA and serum RBP4 in the hypothyroidism group were higher than those in the normal control group (*P* *<* 0.05), as shown in Table 4 and Figure 1.

### 3.5. Multivariate Logistic Regression Analysis of Factors Affecting the Occurrence of Subclinical Hypothyroidism during Pregnancy in Nonobese Pregnant Female

Multivariate logistic regression analysis showed that at age ≥30 years, the increased BPA and RBP4 were the risk factors for subclinical hypothyroidism during pregnancy in the nonobese female, as shown in Table 5.

## 4. Discussion

The thyroid hormone is one of the most important endocrine hormones in the human body and it plays an important role in fetal growth and progression. The fetus cannot produce thyroid hormone in the early stage of pregnancy and it needs to be taken from the mother [7]. Therefore, the thyroid hormone synthesized by the mother during pregnancy is not only for her own needs but also to ensure the needs of the fetus. Any thyroid disease during pregnancy, whether hypothyroidism or hyperthyroidism, can cause various pregnancy complications and cause reversible or irreversible harm to the fetus [8]. Serum FT3, FT4, and TSH are important indicators for evaluating the thyroid function [9]. As a thyroid inhibitory antibody, the change of TPO-Ab concentration is negatively correlated with the secretion of the thyroid gland [10]. The research reports have shown that the TPO-Ab positivity has a certain correlation with the changes in the thyroid hormone levels in pregnant women, and the changes in its levels have a certain role in determining thyroid dysfunction [11]. This study demonstrated that TSH levels in the third trimester were higher than that in early and second trimesters, and the TSH levels in the second trimester were higher than that in early trimesters, while the FT3, FT4, and TPO-Ab levels were lower than that in the early and second trimesters, but in the second trimester, their levels were higher than that in the early trimesters.

BPA is widely used in thermal paper for various purposes such as sealants for dental fillings, medical devices, and containers for the production of food and beverages. The general population in the long-term is mostly exposed to the environmental BPA in low doses [12, 13]. As an endocrine disruptor, BPA has a significant impact on the reproduction of mammals and involves multiple reproductive links such as pregnancy, fertilization, and development [14]. The BPA can enter the human body through the respiratory tract, gastrointestinal tract, and skin and can accumulate in multiple organs and tissues, resulting in potential harm to human health through different molecular mechanisms [15]. In addition, the BPA has fetal toxicity, teratogenicity, and antiandrogen and estrogenoid effect, which can affect the development and reproduction, and is associated with some adverse pregnancy outcomes [16]. RBP-4 is a newly discovered adipocytokine. It can increase insulin levels in both mice and humans, and its low levels can improve insulin sensitivity [17]. At present, the specific mechanism of insulin change caused by RBP-4 has not been fully clarified and there are many studies on the effect of RBP-4 on lipid metabolism and insulin resistance in obese and diabetic patients, while few on hypothyroidism. Insulin resistance and fasting insulinemia have been reported in subclinical hypothyroidism, but their significance has not been well explored [18]. This study showed that the levels of BPA and RBP4 were significantly increased in gestational diabetes mellitus, gestational hypertension, intrahepatic cholestasis of pregnancy, gestational anemia, and preterm delivery; the hypothyroidism group had higher urinary BPA and serum RBP4 levels than the normal control group, which indicated that the levels of urinary BPA and serum RBP4 in a pregnant female with clinical hypothyroidism were significantly increased; the increase of BPA and RBP4 is the risk factor of subclinical hypothyroidism during pregnancy in the nonobese female.

## 5. Conclusion

In summary, BPA and RBP-4 are closely related to the pregnancy outcome of nonobese subclinical hypothyroidism in the pregnant female. The degree of BPA and RBP-4 in adverse pregnancy outcomes is increased, which is a risk factor for nonobese subclinical hypothyroidism.

## Figures and Tables

**Figure 1:** Comparison of urinary BPA and serum RBP4 between the hypothyroidism group and the normal control group. (a) Comparison of urinary BPA between the hypothyroidism group and the normal control group. (b) Comparison of serum RBP4 levels between the hypothyroidism group and the normal control group. Compared with the normal control group,  ^*∗*^*P* *<* 0.05.

**Table 1:** Comparison of thyroid function levels at different stages of pregnancy ($\bar{x}$ ± *s*).

Group	Number of cases	TSH (*μ*g/L)	FT_3_ (pmol/L)	FT_4_ (pmol/L)	TPO-Ab (IU/ml)
First-trimester group	100	0.82 ± 0.14	4.52 ± 0.19	13.87 ± 1.02	17.75 ± 0.73
Second-trimester group	100	1.39 ± 0.27	4.21 ± 0.16	12.73 ± 0.93	16.69 ± 0.82
Third-trimester group	100	1.76 ± 0.38	3.84 ± 0.23	11.18 ± 1.21	14.32 ± 0.68
*F*		283.960	303.403	162.317	554.818
*P* value		<0.001	<0.001	<0.001	<0.001

**Table 2:** Comparison of urinary BPA levels in different pregnancy outcomes ($\bar{x}$ ± *s*).

Pregnancy outcomes	Number of cases	BPA (ng/ml)	*t*	*P* value
*Gestational diabetes*				
*Y*	36	95.42 ± 14.34	27.441	<0.001
*N*	264	47.82 ± 8.98		

Gestational hypertension				
*Y*	47	89.94 ± 12.51	24.199	<0.001
*N*	253	51.32 ± 9.53		

Intrahepatic cholestasis of pregnancy				
*Y*	28	76.42 ± 15.23	5.272	<0.001
*N*	272	64.97 ± 10.42		

Pregnancy anemia				
*Y*	42	82.31 ± 14.32	12.851	<0.001
*N*	258	60.12 ± 9.76		

*Preterm birth*				
*Y*	35	90.12 ± 15.64	22.921	<0.001
*N*	265	50.21 ± 8.62		

**Table 3:** Comparison of serum RBP4 levels in different pregnancy outcomes.

Pregnancy outcomes	Number of cases	RBP4 (*μ*g/L)	*t*	*P* value
*Gestational diabetes*				
*Y*	36	8.10 ± 1.43	11.836	<0.001
*N*	264	6.18 ± 0.82		

*Gestational hypertension*				
*Y*	47	7.96 ± 1.23	11.274	<0.001
*N*	253	6.37 ± 0.81		

*Intrahepatic cholestasis of pregnancy*				
*Y*	28	7.56 ± 1.23	7.904	<0.001
*N*	272	6.08 ± 0.91		

*Pregnancy anemia*				
*Y*	42	7.78 ± 1.30	13.054	<0.001
*N*	258	5.89 ± 0.78		

*Preterm birth*				
*Y*	35	8.04 ± 1.18	11.721	<0.001
*N*	265	5.94 ± 0.97		

**Table 4:** Comparison of urinary BPA and serum RBP4 between the hypothyroidism group and the normal control group ($\bar{x}$ ± *s*).

Group	Number of cases	BPA (ng/ml)	RBP4 (*μ*g/L)
Hypothyroidism group	30	91.42 ± 13.42	7.18 ± 1.09
Normal control group	30	49.58 ± 8.68	5.24 ± 1.31
*T*		14.339	6.235
*P* value		<0.001	<0.001

**Table 5:** Multivariate logistic regression analysis of factors influencing subclinical hypothyroidism during pregnancy in the nonobese female.

Factor	*B*	S.E	*χ* ^2^	*P* value	OR	95% CI
Age ≥30 years	1.451	0.481	9.100	0.003	4.267	1.662∼10.955
Education degree	0.676	0.486	1.935	0.164	1.966	0.758∼5.097
Drinking history	0.737	0.402	3.361	0.067	2.090	0.950∼4.595
Smoking history	0.741	0.452	2.688	0.101	2.098	0.865∼5.088
Folic acid supplementation during pregnancy	0.942	0.604	2.432	0.119	2.565	0.785∼8.380
History of pregnancy and childbirth	0.825	0.528	2.441	0.118	2.282	0.811∼6.423
Abortion history	0.894	0.557	2.576	0.108	2.445	0.821 ∼7.284
Increase of BPA	1.661	0.486	11.681	0.001	5.265	2.031∼13.648
Increase of RBP4	1.657	0.510	10.556	0.001	5.244	1.930∼14.248

## Data Availability

The simulation experiment data used to support the findings of this study are available from the corresponding author upon request.
